# Activation of c-Src tyrosine kinase mediated the degradation of occludin in ventilator-induced lung injury

This article has been retracted.

**DOI:** 10.1186/s12931-014-0158-2

**Published:** 2014-12-04

**Authors:** Tao Zhao, Mengjie Liu, Changping Gu, Xin Wang, Yuelan Wang

**Affiliations:** Department of Anesthesiology, Qianfoshan Hospital, Shandong University, No. 16766 Jingshi Road, Jinan, 250014 Shandong Province China; Department of Anesthesiology, Jinan Fifth People’s Hospital, Ji’nan, Shandong China

**Keywords:** Ventilation-induced lung injury, Tight junctions, Occludin, c-Src inhibitor

## Abstract

**Background:**

Ventilator-induced lung injury (VILI) is characterized by increased alveolar permeability, pulmonary edema. The tyrosine kinase, c-Src, is involved in VILI but its role has not been fully elucidated. This study examined the relationship between c-Src activation and occludin levels in VILI both *in vitro* and *in vivo*.

**Methods:**

For the *in vivo* study, Wistar rats were randomly divided into five groups: control (group C); normal tidal volume (group M); normal tidal volume + c-Src inhibitor (PP2) (group M + P); high tidal volume (group H); and high tidal volume + c-Src inhibitor (PP2) (group H + P). Rats in all groups but group C underwent mechanical ventilation for 4 h. For the *in vitro* study, MLE-12 cells pretreated with PP2 and siRNA underwent cyclic stretching at 8% or 20% for 0, 1, 2 and 4 h. The expressions of occludin, c-Src, and p-c-Src were analyzed by western blotting, hematoxylin and eosin (HE) staining, and immunofluorescence.

**Results:**

For the *in vivo* study, rats in group H showed decreased occludin expression and activated c-Src compared with group C. HE staining and lung injury score showed more severe lung injury and alveolar edema in group H compared with group M and group C. Group H + P had less pulmonary edema induced by the high tidal volume ventilation. For the *in vitro* study, occludin expression decreased and c-Src activation increased as indicated by the phosphorylation of c-Src over time. Consistently, PP2 could restore occludin levels.

**Conclusions:**

Mechanical ventilation can activate c-Src by phosphorylation and increase the degradation of occludin. c-Src inhibitor can ameliorate barrier function and lung injury by up-regulating occludin.

## Background

Ventilator-induced lung injury (VILI) is a common iatrogenic clinical phenomenon in intensive care and anesthesia [1]. VILI can, both *in vivo* and *in vitro*, decrease oxygenation capacity, increase alveolar membrane permeability, and induce secondary pulmonary function damage and acute respiratory distress syndrome [2,3]. Maintaining normal permeability and the integrity of the alveolar membrane could prevent pulmonary edema, and may play a key role in inhibiting or reducing the subsequent development of lung injury [4].

The barrier function of pulmonary epithelial cells plays an important role in maintaining alveolar membrane permeability and preventing the destruction of alveolar epithelial cell junctions, which could lead to acute lung injury and acute respiratory distress syndrome [5-7]. A recent study demonstrated that the expression of the transmembrane protein occludin and the tight junction protein ZO-1 decreased during cyclic mechanical stretching in primary rat cells [8]. The underlying mechanism for how occludin regulates barrier function is not fully understood.

The c-Src family is a family of non-receptor protein tyrosine kinases which regulate cell growth, development, survival and apoptosis, and the regulation of cell or extracellular matrix adhesion functions [9]. The role of c-Src effect on occludin in VILI is unknown.

In this study, we used both *in vivo* and *in vitro* models of VILI to explore the mechanisms behind occludin expression and c-Src and to obtain data that could be used to assist in therapies for the prevention and treatment in VILI.

## Methods

### Materials

Cell culture medium (DMEM/F12) and fetal bovine serum (FBS) were from Gibco. Rabbit c-Src polyclonal antibody (SRC 2) was purchased from Santa Cruz Biotechnology. Rabbit phosphorylation c-Src (Y416) was purchased from CST. The effective and selective inhibitor of c-Src PP2 (172889-27-9) was purchased from Cayman Chemical. Rabbit anti-occludin polyclonal antibody and rabbit anti-GAPDH polyclonal antibody were purchased from Invitrogen. Mouse alveolar epithelial cells (MLE-12) were purchased from American Type Culture Collection (Manassas, VA).

### Cell culture, transient transfection of siRNA and treatment with c-Src inhibitor

MLE-12 cells were plated at a density of 2.5 × 10^5^ cells/ml on culture dishes or BioFlex plates with collagen protein coated in DMEM/F12 and with 10% FBS at 37°C in 5% CO_2_, and incubated for 24–48 h. MLE-12 cell monolayers were serum-deprived for 2 h prior to experiments. For some experiments, PP2 was added to the plate of confluent MLE-12 cells 30 min prior to stretching [10,11].

For transient transfection of Occludin-siRNA, siRNA was synthesized by GenePharma Co., Ltd. (Shanghai, China). The gene sequences are 5′-GCUCUCUCGUCUAGAUAAATT-3′ and 5′-UUUAUCUAGACGAGAGAGCTT-3′. MLE-12 cells were plated at a density of 2.5 × 10^5^ cells/ml on BioFlex plates with collagen protein coated in DMEM/F12 and with 10% FBS at 37°C in 5% CO_2_, and incubated for 24 h before being washed twice with PBS. Then siRNA was diluted with 2 mL DMEM/F12 to remove FBS. INTERFERin (Polyplus-transfection, France), a transfection reagent, was added and eddied for 10 s. The INTERFERin and siRNA dilution was then incubated at room temperature for 10 min before being further incubated at 37°C and 5% CO_2_ for 48 h. Transfection efficiency was measured by western blotting [12,13].

For inhibitor studies, when MLE-12 cell monolayers on BioFlex plates had grown 85–95%, the cells were serum-deprived for 2 h prior to experiments and treated with Src inhibitor PP2 100 nM and DMSO 30 μL/mL for 30 min at 37°C and 5% CO_2_ for cyclic stretching testing [10].

### Cyclic stretching

MLE-12 cells on collagen-coated flexible bottom BioFlex plates were exposed to cyclic stretching using a FX-5000 T Flexercell Tension Plus system (Flexcell International, McKeesport, PA) equipped with a 25-mm BioFlex loading station. After a 48 h culture, cell monolayers were mounted onto the Flexercell system. We used a pattern of cyclic stretching at a frequency 0.5 Hz for 30 cycles/min with a stretch-to-relaxation relation of 1:1 [10,11]. Cyclic stretching was conducted at 8% and 20% of the change in the basement membrane surface area applied in a cyclic manner. These surface area changes correspond to 50% and 80% of total lung capacity, respectively [14,15]. Cyclic stretching time was 1, 2, and 4 h at 37°C in a humidified incubator containing 5% CO_2_. A computer controlled all processes. Non-stretched cells were used as controls. Comparisons were made between stretched cells and control cells cultured on the same plates in the absence of cyclic strain.

### Animals and treatments

Thirty healthy Wistar rats weighing 250–300 g were provided by the Laboratory Animal Center of Shandong Traditional Chinese Medicine University. All animal procedures were reviewed and approved by the Laboratory Animal Ethics Committee of Shandong University.

Rats were randomly divided into five groups (*n* = 6 in each group): a control group (group C); a normal tidal volume group (group M); a normal tidal volume + c-Src inhibitor (PP2) group (group M + P); a high tidal volume group (group H); and a high tidal volume + c-Src inhibitor (PP2) group (group H + P).

Rats in group C did not have mechanical ventilation. The other four groups were mechanically ventilated for 4 h using an ALC-V8 animal ventilator. The tidal volume was 7 mL/kg in group M and group M + P, and 42 mL/kg in group H and group H + P. Ventilation parameters were set as follows: a respiratory rate of 40 times/min, I/E ratio of 1:2, and a fraction of inspired oxygen of 21% [16]. Rats in group M + P and group H + P were pretreated with PP2 1 μg/kg for 1 h before anesthesia.

Animals were anesthetized by intraperitoneal injection of pentobarbital sodium (60 mg/kg) and ketamine (80 mg/kg). Anesthesia was maintained by infusion of pentobarbital at 15 mg/kg every 30 min via the tail vein. Muscle relaxation was maintained with pancuronium (2 mg/kg/h) [17]. Rats’ vital signs were monitored with Mouse Ox pulse oximetry system (Starr Life Sciences Inc, USA).

After ventilation, rats were killed by exsanguination of arterial blood. Lung injury score was recorded [18]. Acute lung injury was scored according to the following four items: alveolar congestion, hemorrhage, infiltration or aggregation of neutrophils in the airspace or the vessel wall, and thickness of the alveolar wall/hyaline membrane formation [18]. Lungs were removed and the right lung upper lobe was quickly frozen in liquid nitrogen which was used for western blotting, and the remnant right lung tissue were fixed in 4% paraformaldehyde for 48–72 h for HE staining. The left lung was used to calculate the pulmonary wet-to-dry (W/D) ratio to quantify the magnitude of pulmonary edema. After measuring the wet lung weight, tissues were incubated in a 70°C incubator for 72 h to gain the dry weight.

### Immunofluorescence and HE staining

For the *in vitro* study, after cyclic stretching, the plates were washed with PBS and cells were fixed in 4% formaldehyde (10 min) and incubated in 1% BSA for 1 h. Cells were then incubated with rabbit anti-occludin polyclonal antibody (1:80 dilution) overnight at 4°C. The secondary antibody (red) was goat anti-rabbit IgG (H + L) used at a 1/150 dilution for 1 h. DAPI was used to stain cell nuclei (blue) for 3 min.

For the *in vivo* study, lung tissues blocked by embedding in paraffin were sectioned and stained with HE staining. Hematoxylin was applied for 5 min and eosin for 2 min.

### Western blotting

For the *in vivo* study, tissue fragments were lysed in radioimmunoprecipitation assay buffer supplemented with a cocktail of protease inhibitors. For the *in vitro* study, for the preparation of total cell extracts, monolayer cultures were washed in cold PBS and lysed in the appropriate amount of RIPA buffer supplemented with the protease inhibitor PMSF. The lysate was collected and protein concentration was determined using a bicinchoninic acid protein assay kit.

Equal amounts of protein were denatured and separated on 10% SDS-PAGE gels and then transferred to polyvinylidene difluoride membranes (Bio-Rad, Hercules, CA, USA) for electrophoresis at 100 V for 1 h.

After blocking with skim milk (5%), proteins were probed overnight at 4°C. Anti-occludin was used at a 1:200 dilution, anti-phosphorylation c-Src at a 1:2000 dilution and anti-c-Src at a 1:1000 dilution. The appropriate horseradish peroxidase-conjugated secondary antibody was added to the filters followed by incubation for 1 h at room temperature with a 1:5000 dilution.

After sequential washing of membranes in T-PBS to remove excess secondary antibody, signals were detected by chemiluminescence using the ECL system. Relative band densities of the various proteins were measured from scanned films using Image J Software.

### Statistical analysis

Representative experiments from at least three independent experiments are shown. Statistical analysis was performed using the SPSS 19.0 statistics package. All data are expressed as mean ± SD. Statistical differences were assessed using Student’s *t*-tests or Tukey and LSD (L) of one-way analysis of variance (ANOVA), where appropriate among groups. A *P*-value <0.05 was considered statistically significant.

## Results

### 8% or 20% cyclic stretching mediated the down-regulation of occludin and the activation of c-Src

MLE-12 cells were treated with 8% or 20% cyclic stretching for 0, 1, 2 and 4 h. Occludin levels and total and phosphorylation of c-Src were detected by western blotting. Occludin expression was not significantly changed at 8% cyclic stretching (*P* > 0.05) (Figure 1). At 20% cyclic stretching, the expression of occludin was reduced in a time-dependent manner, reaching a final reduction of 70% at 4 h (*P* < 0.05) (Figure 1). After exposure of MLE-12 cells to 20% cyclic stretching for 0, 1, 2 and 4 h, c-Src was activated, and the level of total and phosphorylation c-Src increased (*P* < 0.05) (Figure 2).

**Figure 1:** **Time course of cyclic stretch-induced degradation of occludin in MLE-12 cells.** MLE-12 epithelial cells were exposed to 8% or 20% cyclic stretching for 0, 1, 2, and 4 h. Occludin expression was determined by Western blotting. The density of proteins in 0 h was used as a standard (1 arbitrary unit) to compare relative densities in the other times. **P < 0.05,*P < 0.05, compared with 0 h. Data are representative of 3 independent experiments.

**Figure 2:** **Effect of the expressions of total and phosphorylated c-Src on 20% cyclic stretching.** MLE-12 epithelial cells were exposed to 20% cyclic stretching for 0, 1, 2, and 4 h. **A** and **B**: Representative Western blotting of total and phosphorylated c-Src expressions, the density of proteins in 0 h was used as a standard (1 arbitrary unit) to compare relative densities in the other times. *P < 0.05, ^#^ *P* < 0.05, compared with 0 h. Data are representative of 3 independent experiments.

### The c-Src inhibitor PP2 can rescue the cyclic stretching induced occludin loss

MLE-12 cells were randomly divided into four groups: a control group; a stretching group, with 20% cyclic stretching for 4 h; a DMSO group, treated with DMSO for 30 min before stretching; and a PP2 group, pretreated with PP2 for 30 min before stretching. The expression of occludin and c-Src were analyzed by western blotting. The expression of occludin and total and phosphorylation c-Src in the stretching and DMSO groups did not significant change (*P* > 0.05) (Figure 3A,B,C). DMSO used to dilute PP2 was therefore not related to the reduction of occludin or the activation of c-Src. Total and phosphorylated c-Src levels in the PP2 group were lower than those levels in the stretching group (*P* < 0.05) (Figure 3B,C), Occludin levels in the PP2 group were higher than those levels in the stretching group (*P* < 0.05) (Figure 3A), indicating that PP2 can reverse the expression of occludin.

**Figure 3:** **Effect of occludin and c-Src expressions on 20% cyclic stretching with PP2 and DMSO.** MLE-12 cells were exposed on 20% cyclic stretching for 4 h. **A**, **B** and **C**: Representative Western blotting of occludin and total and phosphorylated c-Src expressions and the density of proteins in non-stretching group was used as a standard to compare relative densities in the other groups. *P > 0.05, compared with the DMSO group. **P < 0.05, ^##^ *P* < 0.05, ^#^ *P* < 0.05, compared with the PP2 group. Data are representative of 3 independent experiments. **D**: At the end of cyclic stretching, cells were fixed, blocked and then incubated with occludin primary antibody, performed overnight at 4°C. Cy3-Goat Anti-Rabbit IgG (Red) was used as the secondary antibody. Nuclei were counterstained with DAPI (Blue).

With immunofluorescence, we observed the same distribution of occludin in the stretching and DMSO groups. The distribution of occludin in the stretching group was more limited under microscope than the control group. Compared with the stretching group, occludin distribution in the PP2 group showed a broader scope (Figure 3D).

### The relationship between occludin and c-Src was further confirmed by occludin-siRNA

MLE-12 cells were manipulated at 10 nM, 20 nM and 30 nM concentrations of occludin-siRNA to choose proper concentration for stretching before being examined by western blotting (*P* < 0.05) (Figure 4). c-Src levels did not show significant differences among MLE-12 cells treating with different concentrations of occludin-siRNA (*P* > 0.05) (Figure 5). Compared with MLE-12 cells that had been stretched, the level of c-Src in MLE-12 cells pretreating with Occludin-siRNA did not change (*P* > 0.05) (Figure 5). Knock down of occludin did not appear to affect the expression of c-Src, regardless of whether cells were stretched.

**Figure 4:** **Occluin expression in MLE-12 cells treated by different concentrations of occludin-siRNA.** MLE-12 epithelial cell monolayers were incubated with different concentrations. Representative Western blotting of occludin protein expressions and the density of proteins in occludin-siRNA 0nM group was used as a standard to compare relative densities in the other groups. *P < 0.05, compared with the occludin-siRNA 30 nM group. Data are representative of 3 independent experiments.

**Figure 5:** **Effect of c-Src expression with different treatments in MLE-12 cells.** MLE-12 cells transfected with occludin-siRNA 30 nM were exposed to 20% cyclic stretching for 4 h. Representative Western blotting of c-Src expressions and the density of proteins in non-stretching group was used as a standard (1 arbitrary unit) to compare relative densities in the other groups. *P > 0.05, compared with the non-stretching group. ^#^ *P* > 0.05, compared with the stretching (4 h) group. Data are representative of 3 independent experiments.

### In vivo expression of occludin and c-Src, and pulmonary edema

Mechanical ventilation increased the expression of total and phosphorylation c-Src and the degradation of occludin in group H (*P* < 0.05) compared with group C and M (Figure 6), as seen by western blotting. The expression of occludin was higher and c-Src level was lower in group H + P compared with group H (*P* < 0.05) (Figure 6). HE staining (Figure 7), lung injury score (Table 1) and W/D ratio (Table 2) showed that high tidal volume mechanical ventilation could cause alveolar congestion, infiltration or aggregation of neutrophils in the airspace or the vessel wall, and thickening of the alveolar wall. PP2 could ameliorate the lung injury. These results suggest that high tidal volume mechanical ventilation can activate c-Src and decrease occludin levels.

**Figure 6:** **Expression of occludin and total and phosphorylated c-Src in group C, group M, group M + P, group H and group H + P. A**: Occludin expression was determined by Western blotting analysis and the density of Occludin in control group was used as a standard (1 arbitrary unit) to compare relative densities in the other groups. ^###^ *P* < 0.05, compared with group C. ^##^ *P* < 0.05, compared with group M. ^#^ *P* < 0.05, compared with group H. **B** and **C**: Total and phosphorylation c-Src expressions were determined by Western blotting analysis and the density in control group was used as a standard (1 arbitrary unit) to compare relative densities in the other groups. &&&*P* < 0.05, ***P < 0.05, compared with group C. &&*P* < 0.05, **P < 0.05, compared with group M. &*P* < 0.05, *P < 0.05, compared with group H. Data are representative of 3 independent experiments.

**Figure 7:** **Histological observation of lung injury in group C, group M, group M + P, group H and group H + P.** Lung tissue sections were stained with hematoxylin-eosin (original magnification, ×200). One representative image for each of the lung microscopic photograph in the **(A)** group C, **(B)** group M, **(C)** group M + P, **(D)** group H, **(E)** group H + P, in three independent experiments is shown.

**Table 1:** **Lung injury scores in all groups in vivo**

**Group**	**Alveolar congestion**	**Hemorrhage**	**Infiltration of neutrophils**	**Alveolar wall thickness**	**Total score**
Group C	0	0	0	0	0
Group M	0.33 ± 0.52	0	0.67 ± 0.52	0.5 ± 0.55	1.33 ± 1.51
Group M + P	0.33 ± 0.52	0	0.33 ± 0.52	0.33 ± 0.52	1.00 ± 1.26
Group H	1.67 ± 0.82	0	1.33 ± 0.52	1.5 ± 0.55	4.50 ± 0.84*&
Group H + P	0.50 ± 0.55	0	0.50 ± 0.55	0.67 ± 0.82	1.67 ± 1.21^#^

Data are presented as mean ± SD. *P < 0.05 versus Group C; ^#^ *P* < 0.05 versus Group H; &*P* < 0.05 versus Group M. Lung injury was scored in each sample (n = 6 for each group) according to the following four items: alveolar congestion, hemorrhage, infiltration or aggregation of neutrophils in airspace or the vessel wall, and thickness of the alveolar wall/hyaline membrane formation. Each item was graded according to a 5-point scale: 0, minimal (little) damage; 1, mild damage; 2, moderate damage; 3, severe damage; and 4, maximal damage.

**Table 2:** **Ratio of wet/dry weight in lung**

**Groups**	**Ratio of wet/dry**
Group C	4.12 ± 0.13
Group M	4.65 ± 0.07
Group M + P	4.34 ± 0.04
Group H	5.43 ± 0.14*^,^&
Group H + P	4.64 ± 0.10^#^

Data are presented as mean ± SD. *P < 0.05 versus Group C; ^#^ *P* < 0.05 versus Group H; &*P* < 0.05 versus Group M. Data are representative of 6 independent experiments.

## Discussion

The mechanisms of VILI are intricate, and studies have shown that were related with inflammation and barrier function [19,20]. Processes of inflammation are well known, but barrier function mechanisms require further study. The barrier function comprises tight junctions and adherens junctions. Adherens junctions consist of integral membrane proteins: E-cadherin, β-catenin, p120-catenin, and α-catenin [21]. Tight junctions consist of occludin, the claudin family of proteins, junctional adhesion molecules, and ZO-1, 2, 3 proteins [22].

Mechanical ventilation could damage alveolar barrier function by down-regulating occludin, potentially leading to pulmonary edema [23]. Epithelial and endothelial cells are known to be involved in alveolar barrier function, and the excessive expansion and collapse of cells could damage the integrity of the alveolar membrane, which is the most usual cause of VILI [20].

In the current study, we focused on the role epithelial cells play in barrier function. The current method of stretching alveolar epithelial cells using a stretch machine to simulate lung expansion and contraction is well-recognized [24]. Experiments have confirmed that a stretch area expanded by 8–10% is defined as physiological stretch stimulation, and a stretch area expanded by more than 20–30% as pathological stretch stimulation. Frequency and maximum amplitude of stretching has been reported to change cell permeability and barrier function [25]. In the current *in vitro* study, there was little effect of an 8% cyclic stretching for 4 h on cells. The extension of time also did not change barrier function.

Consistently, we used *in vivo* models of VILI to investigate the relationship between c-Src activation and decreases in occludin levels. Lung tissue in groups with high tidal volume exacerbated pulmonary inflammation and injury. Pathologic changes were serious: alveolar structures deformed, the alveolar septum thickened, infiltration of inflammatory cells increased, and pulmonary edema present. The W/D ratio was higher and the expression of occludin was lower in the VILI models. The c-Src inhibitor PP2 was able to reverse the damage caused, possibly by decreasing the expression of occludin.

Occludin was the first identified transmembrane protein in tight junctions, with a molecular weight of 65 kDa [26]. Recent studies found that occludin plays a key role in barrier function in tight junctions [26,27]. Phosphorylation and endocytosis of occludin could reduce barrier function [28,29]. Cyclic stretching would cause phosphorylation of occludin by c-Src activation in Caco-2 cells [30]. Occludin plays an important role in pulmonary epithelial barrier function [31]. Whether occludin participates in the pulmonary epithelial barrier dysfunction induced by the mechanical stretch remains to be determined. Our study showed the same results in pulmonary epithelial barrier function. The data from the current study indicates that a high tidal volume decreases the expression of occludin *in vivo*, and cyclic stretching showed the same result *in vitro*; with the expression of occludin decreasing gradually.

Activation of c-Src is involved in cell signal transduction and regulating the expression of cell junction proteins [32]. Tyrosine phosphorylation may promote the degradation of junctional proteins from their cytoskeletal anchors [33] and cause endothelial gap formation, resulting in an increase in vascular permeability [34]. c-Src inhibitors could enhance the adhesion function of cells or the extracellular matrix and improve the barrier function of endothelial cells [35]. A previous study showed that increased vascular permeability in mouse lungs ventilated at high airway pressures could be blocked by c-Src inhibitor PP2 [36].c-Src inhibitors play a key role in cyclic stretching, which increases p120-catenin expression, enhances barrier function and reduces intercellular permeability [10]. The effects of c-Src inhibitors on occludin in tight junctions require further study.

The current *in vivo* and *in vitro* studies revealed that both high tidal volume mechanical ventilation and cyclic stretching resulted in the same phenomenon: they could activate the phosphorylation of c-Src and increase the degradation of occludin, and the c-Src inhibitor PP2 could reverse these processes. Immunofluorescence examination showed that the inhibitor improved the distribution of occludin with cyclic stretching; and from HE staining, lung injury score and W/D ratio in rats, it was observed that c-Src inhibitor could ameliorate pulmonary edema and alleviate alveolar hemorrhage, inflammatory cell infiltration and destroyed pulmonary architecture.

Recent studies have reported that occludin and c-Src are involved in VILI [16,37]. Our findings from the current study are consistent with these reports. The effects occludin and c-Src played in VILI, and whether occludin and c-Src are concomitant phenomenon or have a causal relationship remain to be explored. In this study, western blotting showed that high volume mechanical ventilation activated the phosphorylation c-Src and decreased occludin level*,* PP2 could decrease the degradation of occludin *in vitro* and *in vivo*. And *in vitro* MLE-12 cells treated with occludin-siRNA did not result in a change of c-Src with cyclic stretching. That is to say, decreased occludin expression did not affect c-Src activation. There does, however, appear to be a causal relationship by cyclic stretching activating c-Src, which in turn decreases the expression of occluding, but not a concomitant phenomenon or occludin decreased affected the activation of phosphorylated c-Src.

## Conclusions

The results from this study show that VILI down-regulates the expression of the tight junction protein occludin and weakens the epithelial barrier. VILI can activate c-Src and induce a decrease in occludin expression. c-Src inhibitor was able to alleviate the degradation of occludin, strengthen tight junctions and reduce pulmonary edema in VILI. Our results suggest that c-Src may be an important kinase in VILI. Inhibition of c-Src activation may be a novel and effective target for the prevention and treatment of VILI.

## Abbreviations

VILI: Ventilator-induced lung injury
siRNA: Small interfering RNA
HE: Hematoxylin and eosin
FBS: Fetal bovine serum
W/D: Wet-to-dry
BSA: Albumin from bovine serum
DAPI: 4′,6-diamidino-2-phenylindole
RIPA: Radio immunoprecipitation assay
PMSF: Phenylmethanesulfonyl fluoride
SDS: Sodium dodecyl sulfate
PAGE: Polyacylamide gel electrophoresis
ECL: Electrochemiluminescence
ANOVA: Analysis of variance
DMSO: Dimethyl sulfoxide
